This article has been retracted.

# Effects of Remifentanil and Sufentanil Anesthesia on Cardiac Function and Serological Parameters in Congenital Heart Surgery

**DOI:** 10.1155/2021/4650291

**Published:** 2021-12-23

**Authors:** Zhigang Qin, Younian Xu

**Affiliations:** ^1^Surgical Anesthesia Center, TaiKang Tongji (Wuhan) Hospital, Wuhan, Hubei 430000, China; ^2^Department of Anesthesiology, Wuhan Union Hospital, Tongji Medical College, Huazhong University of Science and Technology, Wuhan, Hubei 430030, China

## Abstract

In this study, we have investigated feasibility of remifentanil and sufentanil anesthesia in children with congenital heart disease surgery and its effects on cardiac function and serological parameters. For this purpose, a retrospective study was conducted on 120 children with congenital heart disease who underwent repair of ventricular septum or atrial septum in our hospital, specifically from January 2016 to January 2018, and 60 patients in each group were randomly divided into the control and treatment groups, respectively. The control group was anesthetized with sufentanil, and the treatment group was anesthetized with remifentanil. The heart function, serological indexes, and adverse reactions were observed and compared. We have observed that there was no significant difference in HR levels between these groups (*P* > 0.05), but SDP and DBP values of the two groups were decreased after anesthetic induction (*P* < 0.05). ACH, cortisol, and lactic acid in the treatment group were significantly lower than those in the control group, and the difference was statistically significant (*P* < 0.05). The incidence of bradycardia, nausea and vomiting, hypotension, muscle rigidity, and respiratory depression in the treatment group was 16.67% lower than that in the control group (*P* < 0.05). Remifentanil has less influence on hemodynamics and a better analgesic effect than fentanyl in inhibiting stress response in congenital heart surgery, which provides reference and basis for children congenital heart surgery.

## 1. Introduction

Congenital heart is a disease in which the fetal cardiovascular system is affected by many factors, such as environment and genetics, and the local structure of the heart is malformed or the channels that should be closed are not closed, resulting in abnormal heart and vascular function. Severely, about half of the children will die of serious complications within one year after birth, which threatens the life and health of patients without timely treatment [1, 2]. With the rapid development of anesthesia, effective anesthesia plays a significant role in the successful operation of congenital heart disease. Reducing the use of opioid is crucial to the fast-track anesthesia technology, meanwhile, employing inhalation anesthesia or intravenous anesthesia short-acting drugs. Sufentanil and remifentanil are new opioid receptor agonists. At present, sufentanil is the most widely used synthetic opioid with the best analgesic effect in clinical practice. High doses of sufentanil are used in traditional vascular anesthesia, which has the advantage of stable hemodynamics and good analgesic effect and has prominent disadvantages of long duration of respiratory inhibition [3]. Thus, clarifying the optimal dose of sufentanil can better provide theoretical basis and specific guidance for clinical application [4]. The latest opioid receptor agonist drug remifentanil, which has the advantages of fast acting, short-acting time, and no accumulation during continuous infusion, has been widely used in clinical [5]. Importantly, remifentanil is generally well tolerated with a low incidence of respiratory depression.

In this study, we have investigated the effects of remifentanil and sufentanil anesthesia on cardiac function and serological indexes in congenital heart disease surgery. For this purpose, a retrospective study was conducted on 120 children with congenital heart disease who underwent repair of ventricular septum or atrial septum in our hospital, specifically from January 2016 to January 2018, and 60 patients in each group were randomly divided into the control and treatment groups, respectively. The control group was anesthetized with sufentanil, and the treatment group was anesthetized with remifentanil. The heart function, serological indexes, and adverse reactions were observed and compared. We have observed that there was no significant difference in HR levels between these groups (*P* > 0.05), but SDP and DBP values of the two groups were decreased after anesthetic induction (*P* < 0.05). ACH, cortisol, and lactic acid in the treatment group were significantly lower than those in the control group, and the difference was statistically significant (*P* < 0.05).

The remaining study is organized as follows. In subsequent section, material and methods which were utilized in the proposed setup are described in detail with specific focus on the selection and exclusion criteria for various patients.

## 2. Materials and Methods

### 2.1. Baseline or Experimental Data

The number of clinical samples included in this study was calculated according to the cross-sectional sample size formula: *Q* = 1 − P and *n* = *ta*2PQ/*d*2, where P presents the prevalence of congenital heart disease, *n* is the sample size, and *d* the allowable error, respectively. In addition, *a* = 0.05, and *ta* = 1.96. The minimum sample size obtained by substituting the formula was 110 cases, and a total of 120 cases were included in this study. Based on the random number remainder grouping method, the cases meeting the inclusion criteria were randomly divided into the control group and treatment group, 60 cases in each group. General information of the two groups, such as gender and age, had no effect on this study. The selected patients all correspond with the American Society of Anesthesiologists (ASA) classification and cardiac function classification II-III.

### 2.2. Inclusion and Exclusion Criteria

#### 2.2.1. Inclusion Criteria

The exclusion criteria were as follows: all patients with congenital heart disease in this study accord with the diagnostic criteria for congenital heart disease in expert consensus on interventional treatment of common congenital heart disease in children [6]. Surgical indications correspond with the criteria of surgical indications for congenital heart disease in Chinese expert consensus on surgical treatment of congenital heart disease [7]. The selected patients were conscious and able to express their wishes, 1 month ≤ age ≤13 years old. Endotracheal intubation time >24 h, cardiac output index <3.0 L·min/m^2^, and clinical data of selected patients were complete.

#### 2.2.2. Exclusion Criteria

The exclusion criteria were as follows: patients with respiratory tract infection, myocardial damage or heart failure, mental disorder, and incomplete clinical data; children who died during the observation period or had tracheal intubation removed within 24 h after surgery, patients with severe pulmonary hypertension and patients with poor compliance or severe organ dysfunction; preoperative pulmonary artery systolic pressure ≥50 mmHg; patients with a history of psychosis or depression, epilepsy, aphasia, and dementia; and other patients who cannot express their own wishes. 3 cases were excluded in the control group, and 4 patients were excluded in the observation group.

### 2.3. Methods

Both groups were treated with conventional ventricular septal repair or atrial septal repair. The patients were under preoperative fasting and water for 4-5 hours. Atropines were given 0.02 mg/kg with injected intramuscular 30 min before the induction of surgery to relieve respiratory depression during anesthesia. Midazolam 0.15 mg/kg was given intravenously 5 min before anesthesia to make the patient enter a sedative and lethargic state. Electrocardiogram, blood pressure, heart rate, pulse, and oxygen protection were established, the child's age and weight were calculated, and anesthesia induction was initiated under target-controlled infusion. Both groups were given intravenous midazolam 0.1 mg/kg, propofol 2.5 mg/kg, and vecuronium 0.02 mg/kg. Patients of children in the control group was given sufentanil (specification: 2 ml: 100 *μ*g 10 PCS/box, Yichang Renfu Pharmaceutical Co., Ltd., H20054172) 2 *μ*g/kg and treated with remifentanil (specification: 1 mg: 100 *μ*g 10 tablets/box Jiangsu Nhwa Pharmaceutical Co., Ltd., H20143314) 2 *μ*g/kg in the observation group. After successful intubation, mechanical ventilation was performed on the anesthesia machine. Isoflurane concentration of 1.2% was maintained in both groups. Isoflurane inhalation was discontinued 20 min before the end of operation, and remifentanil and sufentanil were, respectively, stopped postoperatively.

### 2.4. Observation Indicators

1. Cardiac function indicators: the changes of heart rate (HR), diastolic blood pressure (DBP), and systolic blood pressure (SDP) before anesthesia induction (T1), after endotracheal intubation (T2), after skin resection and thoracotomy (T3), and after blockade and opening (T4) were measured in both the groups
2. Serological indicators: the level of acetylcholine, cortisol, and lactic acid before induction of anesthesia (T1) and after endotracheal intubation (T2) were detected in both the groups
3. Adverse reactions: symptoms including bradycardia, nausea and vomiting, decreased blood pressure, muscle rigidity, respiratory depression, and other adverse reactions during awakening were observed in both the groups

### 2.5. Statistical Analysis

The data were calculated by SPSS 25.0 statistical software and presented as mean ± standard deviation. Difference of measurement data was compared and analyzed by the intergroup independent sample *t*-test or repeated measure ANOVA, and the counting data were analyzed through Fisher's exact probability test or *χ*^2^. *P* < 0.05was statistically significant.

## 3. Experimental Results and Observations

As described above, the selected patients were divided into two different groups based on their properties and applicability. These experiments were repeated at least three times to improve accuracy and precision ratio. Both experimental and benchmark datasets were used for analysis purposes.

### 3.1. Comparison of General Data

The independent sample *t*-test indicated no significant difference in gender, average age, body mass index, operation time, anesthesia duration, cardiopulmonary bypass time, and other general information between the two groups (*P* > 0.05), as given in Table 1.

### 3.2. Comparison of Cardiac Function

Compared with the expression before anesthesia induction, the level of HR was not statistically significant between two groups (*P* > 0.05). The values of SDP and DBP in the two groups decreased after anesthesia induction, and the difference was statistically significant (*P* < 0.05), as given in Table 2.

### 3.3. Comparison of Serological Indicators

After anesthesia, serological indexes of patients in the two groups were significantly improved. ACH, cortisol, and lactic acid in the treatment group were significantly lower than those in the control group, and the differences were statistically significant (*P* < 0.05), as given in Table 3.

### 3.4. Comparison of Adverse Reactions

The incidence of bradycardia, nausea and vomiting, decreased blood pressure, muscle rigidity, and respiratory depression in the treatment group was 21.05%, which was significantly higher than that in the control group (7.14%), with statistical difference (*P* < 0.05), as given in Table 4.

## 4. Discussion

Due to the immature compensatory capacity of various organs in children, anesthesia in cardiac surgery has higher requirements. Under the influence of reoperative stress and cardiopulmonary bypass, patients may suffer organ injury again and lead to functional failure [8]. Therefore, ensuring the stability and rapidity of anesthesia induction is of great clinical significance for patients to safely pass the perioperative anesthesia [9]. Ideal surgical narcotic analgesics for children with congenital heart disease should have the following characteristics: strong action, quick effect, stable pharmacokinetics and pharmacodynamics, no biological activity of metabolites, little influence on hemodynamics, and few adverse reactions, and remifentanil is one of these drugs. Studies on the hemodynamics of remifentanil indicate that it possesses the characteristics of rapid clearance at different ages and is independent of cardiac output and liver and kidney functions. Ultrashort clearance half-life determines the rapid recovery of central nervous system and respiratory system functions [10].

Investigate the feasibility of remifentanil and sufentanil in surgical anesthesia of congenital heart disease under equivalent analgesic dose and the effect of remifentanil and sufentanil on cardiac function and serological indexes. The results demonstrated that SDP and DBP values of the two groups were decreased after anesthesia induction, and the serum indexes of the two groups were significantly improved after anesthesia. ACH, cortisol, and lactic acid in the observation group were significantly lower than those in the control group, and the differences were statistically significant (*P* < 0.05). The incidence of bradycardia, nausea and vomiting, decreased blood pressure, muscle rigidity, and respiratory depression in the treatment group was 16.67% obviously lower than that in the control group (6.67%). These results indicate that remifentanil is better than sufentanil in inhibiting stress response in congenital heart disease surgery and has little impact on hemodynamics. Remifentanil is more likely metabolized by nonspecific esters in blood and other tissues and has a strong affinity with *β*-receptors. Bind the solitary tract nucleus and ninth and tenth pair of cranial nerves to suppress the reflex of opioid receptors on the brain nerve which can achieve 23 times the analgesic effect of sufentanil [11–13]. Further study found that there was no bradycardia and hypotension during cardiopulmonary resuscitation after reducing the total amount of remifentanil due to its rapid hydrolytic inactivation. The subsequent resumption of spontaneous breathing allows the patient to be removed early after surgery without causing respiratory depression. However, the increase of blood pressure during endotracheal intubation and surgical stimulation can be inhibited by remifentanil and mainly manifested as dose-dependent decline in blood pressure and heart rate [14, 15]. The effect of using remifentanil commonly occurs dilating blood vessels and slowing heart rate resulting in bradycardia during anesthesia, while the symptoms of bradycardia disappear after anesthesia. Although remifentanil is superior to traditional opioids, standardized analgesia is still needed.

In conclusion, the stress response in congenital heart disease surgery can effectively inhibit after use of remifentanil and has a little effect on hemodynamics. The effect of anesthesia and analgesia effect is better than sufentanil especially, which provides reference and basis for surgical anesthesia of children with congenital heart disease. Remifentanil is widely used in surgical anesthesia of children with congenital heart disease according to the characteristics of safe, effective, and with less complications. However, the research on the application of remifentanil in children's surgical anesthesia remains in infancy, which requires further in-depth research [16].

## 5. Conclusion

In this study, we have investigated feasibility of remifentanil and sufentanil anesthesia in children with congenital heart disease surgery and its effects on cardiac function and serological parameters. For this purpose, a retrospective study was conducted on 120 children with congenital heart disease who underwent repair of ventricular septum or atrial septum in our hospital, specifically from January 2016 to January 2018, and 60 patients in each group were randomly divided into the control and treatment groups, respectively. The control group was anesthetized with sufentanil, and the treatment group was anesthetized with remifentanil. The heart function, serological indexes, and adverse reactions were observed and compared. We have observed that there was no significant difference in HR levels between these groups (*P* > 0.05), but SDP and DBP values of the two groups decreased after anesthetic induction (*P* < 0.05). ACH, cortisol, and lactic acid in the treatment group were significantly lower than those in the control group, and the difference was statistically significant (*P* < 0.05). The incidence of bradycardia, nausea and vomiting, hypotension, muscle rigidity, and respiratory depression in the treatment group was 16.67% lower than that in the control group (*P* < 0.05). Remifentanil has less influence on hemodynamics and a better analgesic effect than fentanyl in inhibiting stress response in congenital heart surgery, which provides reference and basis for children congenital heart surgery.

## Figures and Tables

**Table 1:** Comparison of general data between two groups (*n*, ($\bar{x}$ ±*s*)).

Groups	Sex (male/female)	Age (year)	BMI (kg/m^2^)	Operation time (min)	Anesthesia time (min)	Cardiopulmonary bypass time (min)
Control group (*n*, 57)	33/24	7.63 ± 1.32	27.31 ± 3.67	140.31 ± 3.24	251.25 ± 13.62	51.27 ± 11.23
Observation group (*n*, 56)	35/21	7.62 ± 1.31	27.33 ± 3.25	139.29 ± 2.95	249.27 ± 13.31	53.25 ± 10.82
*χ* ^2^ */t*	0.250	0.040	0.031	1.749	0.781	0.342
*P*	0.617	0.968	0.976	0.083	0.436	0.954

**Table 2:** Comparison of cardiac function between the two groups ($\bar{x}$ ± *s*).

Indicators	Time	Control group (*n*, 57)	Observation group (*n*, 56)	*t*	*P*
HR (beats/min)	T1	107.27 ± 6.14	108.27 ± 6.23	0.859	0.392
	T2	115.23 ± 3.10	110.25 ± 3.82	7.616	<0.001
	T3	109.34 ± 8.25	106.51 ± 2.82	2.431	0.017
	T4	109.24 ± 8.53	111.67 ± 2.24	2.063	0.042
DBP (mmHg)	T1	53.27 ± 8.21	53.21 ± 8.19	0.039	0.969
	T2	48.23 ± 6.30	52.24 ± 9.64	2.622	0.010
	T3	41.26 ± 10.63	47.62 ± 3.66	4.237	<0.001
	T4	34.24 ± 6.72	37.65 ± 5.10	3.035	0.003
SDP (mmHg)	T1	91.27 ± 6.21	92.27 ± 5.86	0.880	0.381
	T2	105.23 ± 3.17	103.25 ± 4.80	3.010	0.003
	T3	88.34 ± 10.21	84.51 ± 2.84	2.706	0.008
	T4	84.24 ± 2.43	81.67 ± 2.25	5.831	<0.001

**Table 3:** Comparison of serological indexes between the two groups ($\bar{x}$ ± *S*).

Groups	ACH (pg/ml)		Cortisol (ng/ml)		Lactic acid (mmol/L)	
	T1	T2	T1	T2	T1	T2
Control group (*n*, 57)	15.34 ± 2.18	45.78 ± 3.32	136.34 ± 10.25	196.51 ± 2.82	0.93 ± 0.10	1.57 ± 0.24
Observatio*n* group (*n*, 56)	15.26 ± 2.63	37.62 ± 3.66	135.26 ± 10.64	182.16 ± 2.81	0.94 ± 0.13	1.13 ± 0.26
*t*	0.176	12.420	0.55	27.090	0.459	9.350
*P*	0.861	<0.001	0.584	<0.001	0.647	<0.001

**Table 4:** Comparison of adverse reactions between the two groups (*n*, (%)).

Groups	Bradycardia	Nausea and vomiting	Blood pressure reduction	Muscle rigidity	Respiratory depression	Adverse reaction rate
Control group (*n*, 57)	2	5	2	1	2	12 (21.05)
Observatio*n* group (*n*, 56)	1	2	1	0	0	4 (7.14)
*χ* ^2^	—	—	—	—	—	4.497
*P*	—	—	—	—	—	0.034

## Data Availability

The datasets used and analyzed during the current study are available from the corresponding author upon request.
